The article "LINC00958 Inhibits Autophagy of Bladder Cancer Cells via Sponge Adsorption of miR-625-5p to Promote Tumor Angiogenesis and Oxidative Stress" was retracted in 2023. Reasons: unreliable results or conclusions; lack of ethics approval or compliance; concerns about the data; concerns about the peer review.

# LINC00958 Inhibits Autophagy of Bladder Cancer Cells via Sponge Adsorption of miR-625-5p to Promote Tumor Angiogenesis and Oxidative Stress

**DOI:** 10.1155/2022/2435114

**Published:** 2022-10-10

**Authors:** Ying Xiao, Tao Wang, Xiao Cheng, Fangwen Liu, You Wu, Limin Ma, Wenguang Li

**Affiliations:** ^1^Department of Urological Surgery, Affiliated Hospital of Nantong University, Nantong, Jiangsu 226001, China; ^2^School of Medicine, Nantong University, Nantong, Jiangsu 226001, China; ^3^Key Laboratory for Neuroregeneration of Jiangsu Province and Ministry of Education, Co-Innovation Center of Neuroregeneration, Nantong University, Nantong, Jiangsu 226001, China; ^4^Department of Pathology, Affiliated Hospital of Nantong University, Nantong, Jiangsu 226001, China

## Abstract

**Objective:**

This study further explored LINC00958's role in promoting tumor angiogenesis (AG) and oxidative stress (OS) development by inhibiting BC cell autophagy through sponge adsorption of miR-625-5p.

**Methods:**

BC patients and healthy controls who visited our hospital between June 2017 and February 2019 were selected as the research group (RG) and the control group (CG), respectively, with a total of 133 study subjects. Peripheral blood LINC00958 and miR-625-5p in both cohorts of participants were detected. Additionally, human bladder transitional cell carcinoma cells (T24 and J82) and human normal urothelial cells (SV-HUC-1) were purchased. Alterations in cell biological behavior were observed after transfecting miR-625-5p-mimics, miR-625-5p-inhibition, and miR-625-5p-NC sequences into these cells, respectively. Besides, ELISA was performed to quantify inflammatory factors (IFs), AG indicators, and OS indexes in cells. Subsequently, a double luciferase reporter (DLR) assay was performed to verify the targeting relationship between LINC00958 and miR-625-5p. Finally, BALB/c-nu nude mice were purchased, and T24 cells transfected with silenced LINC00958 and miR-625-5p expression sequences were used to establish subcutaneous tumors to observe tumor growth and pathological changes.

**Results:**

RG exhibited higher LINC00958 and lower miR-625-5p than CG. LINC00958 and miR-625-5p were strongly linked to myometrial invasion (MI), lymph node metastasis (LNM), distant metastasis (DM), and histology in BC patients, and the increase of LINC00958 and the decrease of miR-625-5p predicted an increased risk of prognostic death in such patients. After miR-625-5p inhibition, the capacity of BC cells to proliferate, invade, and migrate enhanced and the AG, inflammatory response, and OS injury increased, while the apoptosis rate and autophagy ability decreased. The DLR assay revealed inhibited LINC00958WT fluorescence activity by miR-625-5p-mimics, while the biological behavior of BC cells cotransfected with sh-LINC00958 and miR-625-5p-inhibition had no difference with the functions of sh-control and miR-625-5p-NC cotransfected cells. Finally, the nude mouse tumorigenesis experiment showed that the tumor mass, volume, and histopathological features of the sh-LINC00958 group were decreased compared with the sh-control group, while those of the miR-625-5p-inhibition group were increased versus miR-625-5p-NC.

The article "LINC00958 Inhibits Autophagy of Bladder Cancer Cells via Sponge Adsorption of miR-625-5p to Promote Tumor Angiogenesis and Oxidative Stress" was retracted in 2023. Reasons: unreliable results or conclusions; lack of ethics approval or compliance; concerns about the data; concerns about the peer review.

**Conclusions:**

In BC, LINC00958 is highly expressed while miR-625-5p is underexpressed. LINC00958 can inhibit cell autophagy to enhance cell activity; promote OS, inflammation, and AG; and regulate tumor immunity by targeting miR-625-5p, thus participating in the development of BC.

## 1. Introduction

Bladder cancer (BC), as a clinical high-incidence malignancy, is called “two major killers of male urogenital system” together with prostate cancer [1]. BC has a predilection for men aged 50-70 but may occur in all age groups, including children [2]. Bladder urothelial carcinoma, accounting for more than 90% of all BC cases, is the most common type of BC. It is precisely because of the strong migration ability of bladder epithelial cells that BC often has strong metastasis ability [3]. In the face of the great threat posed by BC, a condition with high incidence, strong metastasis, and poor prognosis, exploring and finding an effective and safe means of diagnosis and treatment have become a clinical focus and difficulty.

In the pathogenic research of modern tumor diseases, long-chain noncoding RNAs (lncRNAs) are one of the focuses of attention [4]. In our previous studies, LINC00958 has been found to promote BC cell growth and epithelial-mesenchymal transition via inhibiting the SAPK/JNK axis [5], but the downstream target genes involved in changes in BC cell behavior regulated by LINC00958 remain unclear. Therefore, this study intends to carry out a comprehensive analysis to address this limitation. Through Starbase, an online target gene prediction website, we preliminarily screened the downstream potential target genes of LINC00958, among which miR-625-5p attracted our attention. Located on human chromosome 14q23.3, this gene was first found to have an aberrant expression in the whole genome of cervical cancer and was subsequently confirmed to be of important potential significance in urogenital tumors such as prostate cancer and endometrial cancer [6–8]. Although the direct relationship between miR-625-5p and BC has not been verified yet, some studies have found that miR-625-5p can form a feedback channel with Runx1t1/TCF4 and promote BC progression under the action of RBM24 [9], which also preliminarily reveals the possible close relationship between miR-625-5p and the occurrence and development of BC. Furthermore, Wang et al. and Yang et al. directly pointed out that LINC00958 is able to promote cervical cancer and lung adenocarcinoma cell metastasis by mediating miR-625-5p [10, 11]. Therefore, we speculate that LINC00958 may also participate in the occurrence and development of BC through miR-625-5p. However, no study has yet analyzed the effect of LINC00958 on BC via miR-625-5p. In addition, miR-625-5p was also found to be a gene closely related to placental oxidation [12]. As we all know, in BC, it is confirmed that the occurrence and development of BC are promoted because of severe oxidative stress in urothelial cells [13]. This further illustrates the potential relationship between LINC00958, miR-625-5p, and BC.

The article "LINC00958 Inhibits Autophagy of Bladder Cancer Cells via Sponge Adsorption of miR-625-5p to Promote Tumor Angiogenesis and Oxidative Stress" was retracted in 2023. Reasons: unreliable results or conclusions; lack of ethics approval or compliance; concerns about the data; concerns about the peer review.

Consequently, this study analyzes the role played by LINC00958 and miR-625-5p in BC through experiments to fill in the gap of previous studies, aimed at providing references for a deeper clinical understanding of the pathogenic mechanism of LINC00958 in BC.

## 2. Materials and Methods

### 2.1. Patient Data

BC patients admitted between June 2017 and February 2019 were selected as the research group (RG) for retrospective analysis, with a total of 133 study subjects. According to the inclusion criteria (BC diagnosis by pathological biopsy in our hospital, age range: 18-70 years, and complete medical records), 74 patients with BC were selected. After further screening based on the exclusion criteria (multiple tumors, cardiovascular diseases, autoimmune defects, mental disorders, liver and kidney dysfunction or abnormalities, hospital referrals, and loss to follow-ups), 52 BC patients were finally enrolled. In addition, healthy subjects during the same period were selected as the control group (CG). According to the eligibility criteria (routine physical examination subjects in our hospital, with complete medical records, age range of 18-70 years, normal physical examination results, no major medical history, and willingness to participate in this study), 81 healthy controls were finally included. All the research participants signed the informed consent form by themselves. In order to ensure the reliability of the experimental results, we first compared the clinical baseline data between the two cohorts of subjects included. The results showed no statistical difference in age, sex, and other data between RG and CG (*P* > 0.05, Table 1), suggesting comparability.

### 2.2. qRT-PCR Detection

The blood samples of both cohorts that were routinely examined at admission were used for qRT-PCR detection. We used TRIzol to isolate total RNA from the sample to be tested and then reverse transcribed it into cDNA for PCR reaction under the following conditions that were run for 35 cycles: 95°C/30 s, 95°C/5 s, 65°C/30 s, and 72°C/30 s. Using GAPDH and U6 as internal reference (with primer sequences constructed by American Invitrogen, Table 2), LINC00958 and miR-625-5p expression was calculated by 2^-*ΔΔ*CT^ [14].

The article "LINC00958 Inhibits Autophagy of Bladder Cancer Cells via Sponge Adsorption of miR-625-5p to Promote Tumor Angiogenesis and Oxidative Stress" was retracted in 2023. Reasons: unreliable results or conclusions; lack of ethics approval or compliance; concerns about the data; concerns about the peer review.

### 2.3. Follow-Up for Prognosis

A 36-month follow-up was performed on BC patients. The termination event was death, and the 3-year survival of BC patients was recorded.

### 2.4. Cell Data

Human bladder transitional cell carcinoma T24 and J82 cells and human normal urothelial SV-HUC-1 cells, all supplied by ATCC, were cultured in a 10% fetal bovine serum- (FBS-) supplemented medium under the conditions of 37°C and 5CO_2_. The sh-LINC00958 of targeted silencing LINC00958 and the corresponding negative control sh-control, as well as miR-625-5p mimic sequence (miR-625-5p-mimics), inhibitor sequence (miR-625-5p-inhibition), and negative control group (miR-625-5p-NC), were all constructed by GenePharma and were transfected into T24 and J82 by referring to Lipofectamine 2000 instructions. PCR detected miR-625-5p expression to verify the transfection success rate.

### 2.5. Cell Proliferation Ability Assay

Cells were seeded into 6-well plates with 4 multiple wells set in each group. At 24 h, 48 h, 72 h, and 96 h of culture, CCK-8 solution (10 *μ*L) was added to one well. A microplate reader read the absorbance at 450 nm wavelength, and the growth curve was drawn. Additionally, cells were inoculated into 6-well plates at 200 cells/mL, and 500 *μ*L FBS was added to each well on the 5th day after plate laying. The supernatant was discarded after colony formation was visible to the naked eye. Then, the cells were fixed with 4% paraformaldehyde and stained with 0.1% crystal violet for counting [15].

### 2.6. Cell Invasiveness Ability Assay

Cells (5 × 10^4^ cells/mL) were inoculated in the upper chamber where 300 mL serum-free medium was added, and Matrigel gel was added between the Transwell chambers. The cell culture solution containing 10% FBS was added into the lower chamber. After 24 h of culture, the surface suspended cells were wiped with Q-tips, immobilized, and stained, and the transmembrane cells were counted in 5 randomly selected target fields [16].

### 2.7. Wound-Healing Assay

The cell concentration was adjusted to 4 × 10^5^/mL, and the cells were seeded into 6-well plates. When the growth density reaches 80-90%, a 10 *μ*L pipette tip was used to draw a vertical line in the culture plate. The scratch area was observed 24 h later, and the cell migration rate was calculated as (0 h scratch distance − 24 h scratch distance)/0 h scratch distance × 100% [17].

The article "LINC00958 Inhibits Autophagy of Bladder Cancer Cells via Sponge Adsorption of miR-625-5p to Promote Tumor Angiogenesis and Oxidative Stress" was retracted in 2023. Reasons: unreliable results or conclusions; lack of ethics approval or compliance; concerns about the data; concerns about the peer review.

### 2.8. Protein Relative Expression Detection

RIPA lysed the cells to extract the total protein. After BCA quantification, the protein was transferred to a PVDF membrane by SDS electrophoresis, followed by 10 min of blocking with 5% defatted milk, as well as overnight incubation (4°C) with monoclonal primary antibodies Bax (1 : 1000), cleaved-caspase3 (1 : 1000), cleaved-caspase9 (1 : 1000), LC3-II (1 : 1000), Beclin1 (1 : 1000), p62 (1 : 1000), and GAPDH (1 : 1000). The next day, the membrane was washed and added with the horseradish peroxidase-labeled secondary antibody goat anti-rabbit IgG (1 : 5000). Protein antibodies were purchased from Invitrogen, USA. ECL was used for color development 4 h later. Then, protein bands were scanned for the analysis of relative expression of proteins by TotalLab Quant with *β*-actin as the internal reference. The relative expression level of the target protein was represented by the ratio of the gray value of the target protein to the gray value of the internal reference protein [18]. All antibodies were purchased from Abcam, China.

### 2.9. ELISA

After trypsin lysis, the cells were centrifuged and resuspended. Inflammatory factors (IFs) including interleukin- (IL-) 1*β*, IL-6, and IL-8; angiogenesis- (AG-) related indices vascular endothelial growth factor (VEGF), VEGF receptor 2 (VEGFR2), and epidermal growth factor (EGF); and oxidative stress (OS) markers superoxide dismutase (SOD), malondialdehyde (MDA), and reactive oxygen species (ROS) were detected following ELISA kit instructions.

### 2.10. Double Luciferase Reporter (DLR) Assay

LINC00958's potential downstream target genes were analyzed by Starbase (URL: https://starbase.sysu.edu.cn/). The potential binding site of miR-625-5p was used to construct the LINC00958 3′UTR vector (mutation mode: A/T and G/C exchanged). LINC00958 3′UTR wild-type (WT) and mutant (MUT) plasmids were constructed and cloned into pGL3 luciferase reporter vector, which was subsequently transfected into miR-625-5p-mimics, miR-625-5p-inhibition, and miR-625-5p-NC, respectively. The DLR analysis system calculated the fluorescence expression 24 h later [19].

### 2.11. Animal Information

Twenty BALB/c-nu nude mice supplied by Beijing Vital River Laboratory Animal Technology (Animal License No. SCXK [Beijing] 2021-0006) were raised in cages (three mice per cage) where they were allowed to eat and drink freely.

### 2.12. Establishment of BC Subcutaneous Tumor-Bearing Mice

Mice were randomized into 4 groups, and 4 × 10^6^ T24 cells transfected with sh-control, sh-LINC00958, miR-625-5p-NC, and miR-625-5p-inhibition were injected into the mouse left armpit subcutaneous tissue, respectively. One mouse was selected from each group every 3 days and sacrificed under anesthesia. The whole subcutaneous tumor-bearing tissue was removed for weighing and volume measurement. Nine days later, all the mice were killed, and the tumor-bearing tissues were taken out and fixed with formaldehyde for HE staining [20].

The article "LINC00958 Inhibits Autophagy of Bladder Cancer Cells via Sponge Adsorption of miR-625-5p to Promote Tumor Angiogenesis and Oxidative Stress" was retracted in 2023. Reasons: unreliable results or conclusions; lack of ethics approval or compliance; concerns about the data; concerns about the peer review.

### 2.13. Statistics and Methods

In this study, all experiments were repeated three times. The statistical analysis was carried out by SPSS22.0 software. Count data, denoted by (*n*(%)), was compared by the Chi-squared test between groups. The statistical methods for measurement data denoted by *χ* ± *s* included independent samples *t*-test, one-way ANOVA, and Bonferroni post hoc testing. Correlation analysis was performed by the Pearson correlation coefficient. For patient survival, it was calculated by the Kaplan-Meier method and compared by the Log-rank test. *P* < 0.05 indicated the presence of statistical significance.

## 3. Results

### 3.1. LINC00958 and miR-625-5p Levels in BC

The test showed that the peripheral blood LINC00958 in RG was 3.21 ± 0.41, which was significantly higher than that in CG (*P* < 0.05, Figure 1(a)), while the peripheral blood miR-625-5p in RG (2.05 ± 0.54) was notably lower versus CG (*P* < 0.05, Figure 1(b)). According to Pearson correlation coefficient analysis, peripheral blood LINC00958 and miR-625-5p in RG were significantly and negatively correlated (*P* < 0.05, Figure 1(c)).

### 3.2. Relationship between LINC00958, miR-625-5p, and BC Patients' Clinicopathologic Feature

The comparison identified no statistical differences in LINC00958 and miR-625-5p levels among patients of different ages, genders, and smoking status (*P* > 0.05), indicating no significant correlation between the two genes with the above clinical features. However, in patients with myometrial invasion (MI), lymph node metastasis (LNM), distant metastasis (DM), and high histological grade, LINC00958 was significantly upregulated (*P* < 0.05) while miR-625-5p was underexpressed (*P* < 0.05, Table 3), suggesting a close connection between the two genes and these clinical features.

### 3.3. Prognostic Implications of LINC00958 and miR-625-5p in BC

Ten BC patients died during the 3-year follow-up, with an overall mortality of 20%. The peripheral blood LINC00958 in the dead patients was 3.66 ± 0.33, which was notably upregulated compared with the surviving patients (*P* < 0.05, Figure 2(a)), while miR-625-5p was 1.55 ± 0.38, lower than that in the surviving patients (*P* < 0.05, Figure 2(b)). Taking the median expression levels of the two as the boundary, patients were subdivided into the corresponding high (LINC00958 ≥ 3.21, *n* = 24; miR‐625‐5p ≥ 2.05, *n* = 29) and lower (LINC00958 < 3.21, *n* = 28; miR‐625‐5p < 2.05, *n* = 23) groups of LINC0958 and miR-625-5p. Further, the prognosis survival curve was plotted, which showed that the 3-year total mortality was evidently higher in the high LINC0958 group than in the low LINC0958 group (*P* < 0.05, Figure 2(c)) and higher in the low LINC00958 group versus the high miR-625-5p group (*P* < 0.05, Figure 2(d)).

The article "LINC00958 Inhibits Autophagy of Bladder Cancer Cells via Sponge Adsorption of miR-625-5p to Promote Tumor Angiogenesis and Oxidative Stress" was retracted in 2023. Reasons: unreliable results or conclusions; lack of ethics approval or compliance; concerns about the data; concerns about the peer review.

### 3.4. Impacts of miR-625-5p on BC Cell Biological Behavior

Similarly, it can be seen that miR-625-5p expression in T24 and J82 was 0.99 ± 0.13 and 1.19 ± 0.13, respectively, which was lower compared with SV-HUC-1 (*P* < 0.05, Figure 3(a)). miR-625-5p expression was found to be the highest in the miR-625-5p-mimics group among the three groups, while that in the miR-625-5p-inhibition group was lower compared with the miR-625-5p-NC group (*P* < 0.05, Figure 3(b)), confirming the successful transfection. Subsequently, in the CCK-8 experiment, the miR-625-5p-mimics group exhibited notably lower cell absorbance than the miR-625-5p-inhibition and miR-625-5p-NC groups at 72 h, while the miR-625-5p-inhibition group showed higher absorbance than the miR-625-5p-NC group (*P* < 0.05, Figures 3(c) and 3(d)). Consistent results were found in the cell cloning experiment, namely, the cell cloning rate of the miR-625-5p-mimics group was the lowest among the three groups, while that of the miR-625-5p-inhibition group was higher as compared to the miR-625-5p-NC group (*P* < 0.05, Figure 3(e)). Finally, in the Transwell experiment, we can see that the number of membrane-penetrating cells in the miR-625-5p-mimics group was 32.67 ± 4.16, 29.33 ± 5.86, significantly lower than that in the other two groups, while the number of membrane-penetrating cells in the miR-625-5p-inhibition group was 163.00 ± 9.54, 172.67 ± 11.50, higher compared with the miR-625-5p-NC group (*P* < 0.05, Figure 3(f)). The cell scratch-wound test results showed a lower cell migration rate in the miR-625-5p-mimics group compared with the other two groups and a higher migration rate in the miR-625-5p-inhibition group versus the miR-625-5p-NC group (*P* < 0.05, Figure 3(g)). Moreover, apoptosis rates were found to be the highest in the miR-625-5p-mimics group among the three groups, while those in the miR-625-5p-inhibition group were lower compared with the miR-625-5p-NC group (*P* < 0.05, Figure 3(h)).

### 3.5. Impacts of miR-625-5p on Immunity and Autophagy of BC Cells

ELISA results showed lower MDA, ROS, IL-1*β*, IL-6, IL-8, VEGF, VEGFR2, and EGF levels while higher SOD levels in the miR-625-5p-mimics group compared with the other two groups (*P* < 0.05); when compared to the miR-625-5p-NC group, MDA, ROS, IL-1*β*, IL-6, IL-8, VEGF, VEGFR2, and EGF were higher in the miR-625-5p-inhibition group, and SOD was lower (*P* < 0.05, Figures 4(a)–4(c)). Further, the detection of autophagy proteins revealed that LC3-II, Beclin1, and p62 in the miR-625-5p-mimics group were 0.87 ± 0.08, 1.01 ± 0.07, and 0.92 ± 0.06, respectively, which were the highest among the three groups, while the data in the miR-625-5p-inhibition group were 0.12 ± 0.03, 0.08 ± 0.06, and 0.10 ± 0.02, respectively, which were the lowest (*P* < 0.05, Figures 4(d) and 4(e)).

The article "LINC00958 Inhibits Autophagy of Bladder Cancer Cells via Sponge Adsorption of miR-625-5p to Promote Tumor Angiogenesis and Oxidative Stress" was retracted in 2023. Reasons: unreliable results or conclusions; lack of ethics approval or compliance; concerns about the data; concerns about the peer review.

### 3.6. Verification of Targeting Relationship between LINC00958 and miR-625-5p

We found through Starbase the binding complementary loci between LINC00958 and miR-625-5p (Figure 5(a)), so we further used the DLR assay to validate the relationship between the two genes. The results determined that the LINC00958-WT fluorescence activity after miR-625-5p-mimics transfection was 0.35 ± 0.07, which was obviously lower compared with that after miR-625-5p-NC transfection (*P* < 0.05), while after miR-625-5p-inhibition transfection, the fluorescence activity of LINC00958-MUT increased obviously (*P* < 0.05, Figure 5(b)), indicating a targeted regulatory relationship between the two. After transfection of SH-LINC00958 into T24 and J82, miR-625-5p levels in these cells were markedly upregulated compared with sh-control transfected cells (*P* < 0.05, Figure 5(c)).

### 3.7. LINC00958 Affects BC Cell Biological Behavior via Sponge Adsorption of miR-625-5p

Cells with different transfections were grouped as follows: group A: sh-control+miR-625-5p-NC, group B: sh-control+miR-625-5p-inhibition, group C: sh-LINC00958+miR-625-5p-NC, group D: sh-LINC00958+miR-625-5p-inhibition, and group E: sh-LINC00958. Then, the biological behaviors of the above groups of cells were examined. First of all, CCK-8 and cell cloning experiments showed that the cell optical density and cloning rate of group B were the highest among the five groups; no evident differences were found between groups A and D and between groups C and E (*P* > 0.05), among which groups C and E had lower cell optical density and cloning rate than groups A and D (*P* < 0.05, Figures 6(a)–6(c)). Groups A and D also showed a similar number of membrane-penetrating cells and cell mobility (*P* < 0.05), lower than those in group B (*P* < 0.05). Nor were there any notable differences between groups C and E in the number of membrane-penetrating cells and cell mobility (*P* > 0.05), which were lower compared with groups A and D (*P* < 0.05, Figures 6(d) and 6(e)). Finally, the detection results of the apoptotic rate were the lowest in group B and highest in groups C and E, while their levels in groups A and D were higher compared with group B and lower compared with groups C and E (*P* < 0.05, Figure 6(f)).

The article "LINC00958 Inhibits Autophagy of Bladder Cancer Cells via Sponge Adsorption of miR-625-5p to Promote Tumor Angiogenesis and Oxidative Stress" was retracted in 2023. Reasons: unreliable results or conclusions; lack of ethics approval or compliance; concerns about the data; concerns about the peer review.

### 3.8. LINC00958 Affects Immunity and Autophagy in BC Cells via Sponge Adsorption of miR-625-5p

In subsequent tests, it was found that the conditions of the five groups of cells were basically consistent with the abovementioned biological behaviors; that is, there was no difference in all test results between groups A and D and between groups C and E (*P* > 0.05). Among them, MDA, ROS, IL-1*β*, IL-6, IL-8, VEGF, VEGFR2, and EGF in groups A and D were lower versus group B and higher versus groups C and E (*P* < 0.05); on the contrary, SOD in groups A and D was higher compared with group B and lower versus groups C and E (*P* < 0.05, Figures 7(a)–7(c)). Similarly, autophagy proteins LC3-II, Beclin1, and p62 in groups A and D were lower compared with groups C and E, but higher than those in group B (*P* < 0.05, Figures 7(d) and 7(e)).

### 3.9. Impacts of LINC00958 and miR-625-5p on Tumorigenesis

First, comparing the tumor-bearing growth of mice in each group (Figure 8(a)), it was found that the tumor mass and volume in the sh-LINC00958 group were markedly lower compared with the sh-control group (*P* < 0.05, Figures 8(b) and 8(c)), while those in the miR-625-5p-inhibition group were higher versus the miR-625-5p-NC group (*P* < 0.05, Figures 8(d) and 8(e)). HE staining exhibited that the sh-control and miR-625-5p-NC groups had relatively few cells with small nuclei and few cytokinesis and mitosis but showed relatively more necrotic cells and neutrophil and lymphocyte infiltration. Compared with the sh-control and miR-625-5p-NC groups, the tumor tissue of the sh-LINC00958 group was significantly improved, with more dense cells and rich cytoplasm, increased mitosis, and decreased inflammatory cell infiltration. The tumor tissue damage in the miR-625-5p-inhibition group was the most serious, with a large number of cells showing pyknosis and necrosis, and the infiltration of neutrophils/lymphocytes was extremely serious (Figure 8(f)). Therefore, lowering LINC00958 can inhibit BC growth, while reducing miR-625-5p can promote BC growth.

## 4. Discussion

In modern clinical research, it is agreed that the breakthrough in the diagnosis and treatment of neoplastic diseases lies in miRNAs due to their following advantages: (1) they can be conveniently detected in human blood, body fluids, tissues, cells, and other samples; (2) the quantitative analysis results are more objective and accurate, allowing them to be excellent and potential tumor markers [21]; and (3) due to the regulation and influence of miRNAs on the cell life cycle, they can be molecular therapeutic targets for tumors in the future to achieve the purpose of killing tumor cells, thus overcoming the problem that tumors are difficult to completely cure at present [22]. In the previous research, we have clarified the mechanism of LINC00958 in BC [5], but there are still two unsolved problems. First, no clinical tests have been carried out, resulting in the inability to determine the clinical expression of LINC00958 in BC. Second, the downstream target genes involved in LINC00958 regulation of BC cell activity remain to be explored. In view of the above two problems, this study launched a more comprehensive and complete analysis to address its limitations.

The article "LINC00958 Inhibits Autophagy of Bladder Cancer Cells via Sponge Adsorption of miR-625-5p to Promote Tumor Angiogenesis and Oxidative Stress" was retracted in 2023. Reasons: unreliable results or conclusions; lack of ethics approval or compliance; concerns about the data; concerns about the peer review.

First of all, we screened the potential downstream target genes of LINC00958 and initially focused on miR-625-5p based on the results of previous studies. Our clinical examination results showed upregulated LINC00958 and underexpressed miR-625-5p in BC patients, indicating an inverse connection between the two genes in BC. This is consistent with the results of our previous research and related studies [23, 24], confirming that LINC00958 is involved in the occurrence and development of BC and that its mechanism of action may be bound up with miR-625-5p. In the subsequent analysis of the relationship between them and clinical pathology of BC patients, the two genes were found to have a close connection with MI, LNM, DM, and histological grade of BC, which once again verifies our view. This is in consistence with our expectation, as we have confirmed through previous studies that overexpressed LINC00958 in BC can promote the ability of tumor cells to proliferate and invade [5]. While the relationship between miR-625-5p and BC clinicopathological features can further confirm the involvement of miR-625-5p in BC. In the prognostic follow-up, higher LINC00958 and lower miR-625-5p were determined in the surviving patients than in the dead. Further, the prognosis survival curve showed that both the increase of LINC00958 and the decrease of miR-625-5p predicted an increased risk of death in BC patients. It also suggests the potential of the two genes to become the prognostic markers of BC in the future, which can assist clinicians to understand the prognosis of BC patients more quickly, so as to carry out the targeted intervention in a more timely manner to provide more reliable security for patients. The expression in tissues is reported to be more accurate [25], while the clinical analysis in this study was conducted based mainly on blood samples due to the convenience of obtaining blood samples. Hence, LINC00958 and miR-625-5p in BC tissues and adjacent tissues should be detected for validation in the follow-up experiments.

The article "LINC00958 Inhibits Autophagy of Bladder Cancer Cells via Sponge Adsorption of miR-625-5p to Promote Tumor Angiogenesis and Oxidative Stress" was retracted in 2023. Reasons: unreliable results or conclusions; lack of ethics approval or compliance; concerns about the data; concerns about the peer review.

*In vitro*, we also found decreased miR-625-5p in BC cells. After suppressing miR-625-5p, the ability of BC cells to proliferate, invade, and migrate was found to be enhanced, and the apoptosis ability was decreased, but the reverse was true after the expression of miR-625-5p was increased. Thus, miR-625-5p with low expression in BC can also promote BC cell activity and accelerate the malignant progression of BC. Referring to past literature, we also found that the low expression of miR-625-5p can promote glioma invasion and the pathological process of gastric cancer [26, 27], which can also verify the accuracy of the results of this experiment. Besides, OS, inflammation, AG, and tumor immunity are all important pathological changes in the immune studies of BC progression [28–30]. In a study on tumor microcirculation, inhibiting the above reaction processes is also regarded as one of the reliable ways to curb tumor development [31]. Therefore, we also explored alterations in OS, inflammatory responses, AG, and tumor immunity of BC cells under the influence of miR-625-5p. Consistently, miR-625-5p inhibition was accompanied by promoted OS injury, inflammation, AG, and tumor immunity changes of cells, while increasing miR-625-5p inhibited these changes. It also demonstrates the potential of miR-625-5p as a therapeutic target for BC, with great significance in future clinical applications. Autophagy is an evolutionarily conserved and important process for the turnover of intracellular substances in eukaryotes; in tumor cells, autophagy can be activated to induce cell death, which is hailed as the key to future molecular targeted therapy [32, 33]. Existing evidence shows that the autophagy ability of cells is obviously inhibited in BC and can be reactivated via increasing miR-625-5p [34, 35], which validates our view. From this, we can definitely know that miR-625-5p, which is underexpressed in BC, can participate in the development of BC by inhibiting autophagy, enhancing cell activity, regulating tumor immunity, and promoting OS responses, inflammation, and AG.

Finally, we used the DLR assay to verify the relationship between the two genes. The results identified that LINC00958-WT and MUT fluorescence activities were affected by miR-625-5p, and miR-625-5p expression in BC cells was increased after LINC00958 was inhibited, which was consistent with the above clinical examination results, confirming that LINC00958 negatively and targeted modulated miR-625 in BC. Through the rescue experiment, we also found reduced cell OS reaction, inflammatory responses, and AG and activated autophagy after inhibiting LINC00958, further demonstrating the important influence of LINC00958 on BC. Furthermore, cotransfection of LINC00958+miR-625-5p into cells resulted in similar cell biological behavior and pathological changes to those with sh-control+miR-625-5p-NC cotransfection, indicating that miR-625-5p completely reversed the effect of inhibiting LINC00958 on BC cells. Moreover, the cells cotransfected with sh-LINC00958 and miR-625-5p-NC were basically the same as those transfected with sh-LINC00958 alone, confirming that LINC00958 participates in various functional changes of BC cells by targeting miR-625-5p. In the nude mouse tumorigenesis experiment, we also found obviously inhibited tumor growth and improved pathological changes after silencing LINC00958, while completely opposite results were observed following miR-625-5p silencing. These results not only verified the influence of LINC0958 and miR-625-5p on living BC tumors but also preliminarily revealed the significance of LINC0958 and miR-625-5p, which may be therapeutic targets that contribute to a breakthrough for future diagnosis and treatment of BC.

The article "LINC00958 Inhibits Autophagy of Bladder Cancer Cells via Sponge Adsorption of miR-625-5p to Promote Tumor Angiogenesis and Oxidative Stress" was retracted in 2023. Reasons: unreliable results or conclusions; lack of ethics approval or compliance; concerns about the data; concerns about the peer review.

### 4.1. Limitations

Due to the short study period, the small number of cases included in this study, and the relatively short follow-up time, we have been unable to assess the long-term prognosis of patients. Second, we should also verify the effect of LINC00958 and miR-625-5p on the prognosis of BC patients by COX analysis. Finally, we should collect cancerous and paracancerous tissues from BC patients as test samples to confirm the expression of LINC00958 and miR-625-5p, as tissue samples are more accurate than blood samples for PCR experiments. These are the limitations of this study, which will be addressed through future supplementary research.

## 5. Conclusion

LINC00958 was highly expressed in BC, and miR-625-5p was underexpressed. LINC00958 is involved in BC by targeting miR-625-5p to inhibit cell autophagy, enhance cell activity, regulate tumor immunity, and promote OS, inflammation, and AG. Both genes are of great significance to the diagnosis and treatment of BC and are expected to be a breakthrough in the clinical treatment of BC.

## Figures and Tables

**Figure 1:** LINC00958 and miR-625-5p levels in BC: (a) comparison of peripheral blood LINC00958 between the research group (*n* = 52) and the control group (*n* = 81); (b) comparison of peripheral blood miR-625-5p between the research group (*n* = 52) and the control group (*n* = 81); (c) correlation between peripheral blood LINC00958 and miR-625-5p in the research group (*n* = 52). ^#^*P* < 0.05.

The article "LINC00958 Inhibits Autophagy of Bladder Cancer Cells via Sponge Adsorption of miR-625-5p to Promote Tumor Angiogenesis and Oxidative Stress" was retracted in 2023. Reasons: unreliable results or conclusions; lack of ethics approval or compliance; concerns about the data; concerns about the peer review.

**Figure 2:** Prognostic implications of LINC00958 and miR-625-5p in BC: (a) comparison of LINC00958 between dead patients (*n* = 10) and surviving patients (*n* = 42); (b) comparison of miR-625-5p between dead patients (*n* = 1) and surviving patients (*n* = 42); (c) the 3-year survival curve of the high (*n* = 24) and low (*n* = 28) LINC00958 groups; (d) the 3-year survival curve of the high (*n* = 29) and low (*n* = 23) miR-625-5p groups. ^#^*P* < 0.05.

**Figure 3:** Impacts of miR-625-5p on BC cell biological behavior (*n* = 3): (a) comparison of miR-625-5p expression among T24, J82, and SV-HUC-1; (b) PCR verification of transfection success rate of miR-625-5p-mimics, miR-625-5p-NC, and miR-625-5p-inhibition; (c, d) CCK-8 assay was used to detect the effect of miR-625-5p on the growth of T24 and J82 cells; (e) clonal formation experiment was used to detect the effect of miR-625-5p on the proliferation of T24 and J82 cells; (f) Transwell assay was used to detect the influence of miR-625-5p on the invasiveness ability of T24 and J82 cells (200x); (g) cell scratch assay was used to detect the influence of miR-625-5p on the migration ability of T24 and J82 cells; (h) flow cytometry assay was used to detect the influence of miR-625-5p on the apoptotic ability of T24 and J82 cells. Compared with miR-625-5p-NC group (^#^*P* < 0.05); compared with miR-625-5p-mimics group (^&^*P* < 0.05).

**Figure 4:** Impacts of miR-625-5p on immunity and autophagy of BC cells (*n* = 3): (a) impact of miR-625-5p on BC oxidative stress; (b) impact of miR-625-5p on inflammatory responses of BC; (c) impact of miR-625-5p on BC angiogenesis; (d) impact of miR-625-5p on T24 autophagy; (e) impact of miR-625-5p on J82 autophagy. Compared with miR-625-5p-NC group (^#^*P* < 0.05); compared with miR-625-5p-mimics group (^&^*P* < 0.05).

**Figure 5:** Verification of targeting relationship between LINC00958 and miR-625-5p (*n* = 3): (a) binding complementary loci of LINC00958 and miR-625-5p; (b) DLR assay; (c) impact of LINC00958 on miR-625-5p expression. ^#^*P* < 0.05.

**Figure 6:** LINC00958 affects BC cell biological behavior via sponge adsorption of miR-625-5p (*n* = 3): (a, b) CCK-8 experiment detects the growth ability of T24 and J82 cells; (c) the clone formation test detects the proliferation ability of T24 and J82 cells; (d) Transwell assay detects the T24 and J82 cell invasion ability (200x); (e) cell scratch assay detects the T24 and J82 cell migration ability; (f) flow cytometry detects the T24 and J82 cell apoptosis rate. Compared with group A (^#^*P* < 0.05); compared with group B (^&^*P* < 0.05); compared with group C (^@^*P* < 0.05); compared with group D (^∗^*P* < 0.05).

The article "LINC00958 Inhibits Autophagy of Bladder Cancer Cells via Sponge Adsorption of miR-625-5p to Promote Tumor Angiogenesis and Oxidative Stress" was retracted in 2023. Reasons: unreliable results or conclusions; lack of ethics approval or compliance; concerns about the data; concerns about the peer review.

**Figure 7:** LINC00958 affects immunity and autophagy in BC cells via sponge adsorption of miR-625-5p: (a) oxidative stress response in BC cells; (b) inflammatory response in BC cells; (c) angiogenic capacity of BC cells; (d) autophagy capacity in T24; (e) autophagy capacity in J82. Compared with group A (^#^*P* < 0.05); compared with group B (^&^*P* < 0.05); compared with group C (^@^*P* < 0.05); compared with group D (^∗^*P* < 0.05).

**Figure 8:** Impacts of LINC00958 and miR-625-5p on tumorigenesis: (a) the results of the tumorigenesis test in nude mice; (b, c) impacts of LINC00958 on tumorigenesis; (d, e) impacts of miR-625-5p on tumorigenesis; (f) HE staining of tumor tissue sections (100x). ^#^*P* < 0.05.

**Table 1:** Comparison of clinical baseline data.

	Research group (*n* = 52)	Control group (*n* = 81)	*t* or *χ*^2^/*P*
Age	61.33 ± 5.96	62.36 ± 5.40	1.031/0.305
Sex			
Male	47 (90.38)	72 (88.89)	0.075/0.784
Female	5 (9.62)	9 (11.11)	
Smoking			
Yes	37 (71.15)	65 (80.25)	1.465/0.226
No	15 (28.85)	16 (19.75)	
Myometrial invasion			
Yes	15 (28.85)	—	
No	37 (71.15)	—	
Lymph node metastasis			
Yes	13 (25.00)	—	
No	39 (75.00)	—	
Distant metastasis			
Yes	11 (21.15)	—	
No	41 (78.85)	—	
Histological grading			
High	11 (21.15)	—	
Middle	9 (17.31)	—	
Low	32 (61.54)	—	

**Table 2:** Primer sequences.

	F (5′-3′)	R (5′-3′)
LINC00958	CAGCGAAAGGCAGCTGATTC	ATAAAGTGGTCTGGGCCTGC
GAPDH	GAAGGTGAAGGTCGGAGTC	GAAGATGGTGATGGGATTTC
miR-625-5p	GGGGAGGGGGAAAGTTCTA	GTGCGTGTCGTGGAGTCG
U6	GCTTCGGCAGCACATATACTAAAAT	CGCTTCACGAATTTGCGTGTCAT

**Table 3:** Relationship between LINC00958, miR-625-5p, and BC patients' clinicopathologic feature.

	*n*	LINC00958	*t* or *F*/*P*	miR-625-5p	*t* or *F*/*P*
Age	<61 years old	3.18 ± 0.35	0.512/0.611	2.09 ± 0.41	0.390/0.698
	≥61 years old	3.24 ± 0.46		2.03 ± 0.63	
Sex	Male	3.20 ± 0.42	0.724/0.355	2.05 ± 0.57	0.230/0.819
	Female	3.27 ± 0.41		2.11 ± 0.33	
Smoking	Yes	3.23 ± 0.44	0.497/0.621	2.04 ± 0.60	0.372/0.711
	No	3.17 ± 0.35		2.08 ± 0.40	
Myometrial invasion	Yes	3.57 ± 0.36	4.765/<0.001	1.65 ± 0.48	3.880/<0.001
	No	3.07 ± 0.34		2.22 ± 0.48	
Lymph node metastasis	Yes	3.60 ± 0.35	4.639/<0.001	1.54 ± 0.39	4.684/<0.001
	No	3.08 ± 0.35		2.23 ± 0.48	
Distant metastasis	Yes	3.73 ± 0.29	6.186/<0.001	1.54 ± 0.41	4.029/<0.001
	No	3.07 ± 0.32		2.19 ± 0.49	
Histological grading	High	3.70 ± 0.32	15.060/<0.001	1.49 ± 0.34	12.630/<0.001
	Middle	3.43 ± 0.33		1.98 ± 0.43	
	Low	2.98 ± 0.26		2.27 ± 0.48	

## Data Availability

The datasets used and/or analyzed during the current study are available from the corresponding authors on reasonable request.
